# Complement family member CFI polymorphisms and AMD susceptibility from a comprehensive analysis

**DOI:** 10.1042/BSR20200406

**Published:** 2020-04-09

**Authors:** Qianqian Yu, Jing Zhu, Yong Yao, Chao Sun

**Affiliations:** Department of Ophthalmology, Affiliated Wuxi People’s Hospital of Nanjing Medical University, Wuxi, Jiangsu, China

**Keywords:** age-related macular degeneration, complement factor I, meta-analysis, polymorphism, risk

## Abstract

The complement factor I (*CFI*) gene polymorphisms have been reported to age-related macular degenerative (AMD) risk, nevertheless, above association is not consistent. We investigated a meta-analysis to evaluate the conclusions between *CFI* polymorphisms (rs10033900 and rs2285714) and AMD risk. An identification was covered with the PubMed and other databases through February 8, 2020. Odds ratios (OR) and 95% confidence intervals (CI) were used to assess the strength of associations. After a comprehensive search, 11 different articles (12 case–control studies for total AMD and 11 case–control studies about neovascular disease/geographic atrophy in AMD) were retrieved. Individuals carrying C-allele or CC genotype of rs10033900 polymorphism may have a decreased risk to be AMD disease. For example, there has a significantly decreased relationship between rs10033900 polymorphism and AMD both in the whole group, Caucasian population and population-based source of control. Moreover, a similar trend in subgroup of genotype method group by MALDI-TOF MS was detected. To classify the type of AMD in further, decreased association was also observed in both neovascular disease and geographic atrophy AMD. No association was found about rs2285714 polymorphism. Our present groundbreaking study suggests that the *CFI* rs10033900 polymorphism is potentially associated with the risk of AMD development.

## Introduction

Age-related macular degeneration (AMD) is a retinal degenerative disease that is an important cause of blindness and central vision loss in the elderly who are over 55 years [1,2]. The incidence rate is 13%, accounting for 20% of the causes of blindness in the elderly, especially in developed countries [3,4]. The early stages, characterized by subretinal deposits (drusen) on the Bruch membrane and the extracellular matrix separating the choriocapillaris from the retinal pigment epithelium (RPE), affect 15.4% of those aged more than 65 years; the late stages, including abnormal blood vessels growing from the choriocapillaris through the Bruch membrane (neovascular disease or wet AMD) and the degeneration of photoreceptors and RPE cells resulting in geographic atrophy (geographic atrophy or dry AMD) [5]. The exact etiology of AMD has not been determined so far, which is likely to be the result of a complex cross-reflection of multiple factors, such as inheritance, age, ethnicity, family history, smoking, nutritional factors and sun exposure [1,6,7]. A genome-wide association study (GWAS) showed a clearer view about significant links between AMD risk and genetic variations in 2005, suggesting AMD is a polygenic disease [8], which triggered numerous studies involving the genetic associations of AMD in the following 1.5 decades [9–11].

The complement system is an important mediator of natural and acquired immunity in humans [12]. A dysfunctional complement pathway has been proposed to increase retinal cell damage via increased formation of drusen deposits, atrophy, and cell degeneration and progression to choroidal neovascularization (CNV) [13,14]. So far, *component 2* (rs547154 and rs9332739) [15], *component 5* [16], *factor B* (L9H) [17] and *factor H* (Y402H) [18] polymorphisms have been observed associated with AMD susceptibility. In 2015, our team first reported the association between *component 3* gene polymorphisms and AMD risk and suggested rs2230199, rs11569536, rs1047286 and 2250656 SNPs may be related to AMD development [19]. Nowadays, many recent studies focused on another family member in complement system, named factor I (CFI).

CFI gene encodes a serine proteinase that is essential for regulating the complement cascade and is expressed by hepatocytes, macrophages, lymphocytes, endothelial cells and fibroblasts [20]. The encoded preproprotein is cleaved to produce both heavy and light chains, which are linked by disulfide bonds to form a heterodimeric glycoprotein. This heterodimer can cleave and inactivate the complement components C4b and C3b, and it prevents the assembly of the C3 and C5 convertase enzymes [21] (https://www.ncbi.nlm.nih.gov/gene/3426).

Three common polymorphisms in *CFI* gene is rs10033900 (wide allele T to mutation allele C), rs2285714 (wide allele T to mutation allele C) and rs141853578 (wide allele C to mutation allele T). Fagerness et al. first found rs1003390 SNP remained the most highly associated SNP with a *P*-value of 6.46 × 10^−8^ (OR = 0.7056 referring to lower-risk C-allele) for AMD [22]. Subsequently, several related articles have been published.

In view of the foregoing, we realized the vital role of *CFI* gene two common polymorphisms (rs10033900 and rs2285714) and preformed a comprehensive meta-analysis to make convincing conclusions [23–33].

## Methods

### Search strategy

We searched relative studies from PubMed and Other databases (Embase, Google Scholar, Wanfang, CNKI, Web of Science) before February 8, 2020. The keywords were “age-related macular degeneration or AMD,” “polymorphism or variant,” and “CFI or complement factor I.” With these terms, a total of 11 different articles were included from above databases based on our inclusion criteria. Stages of AMD were assigned based on the classification of the Age-Related Eye Disease Study (AREDS) [34].

### Inclusion and exclusion criteria

Included studies were according with (a) the correlation between AMD risk and *CFI* gene rs10033900 and/or rs2285714 polymorphisms; (b) case–control studies, and (c) adequate numbers of each genotypes (CC, CT, and TT) in case and control groups. Studies were excluded if they (a) included no control information; (b) didn't contain genotype frequency data, and (c) were duplicated studies with some other papers.

### Data extraction

Two authors (Qianqian Yu and Chao Sun) independently screened all papers that according with the selection criteria. These data included the first author’s last name, publication year, country of origin, ethnicity, Hardy–Weinberg equilibrium (HWE) of control group, genotyping method and AMD disease types (neovascular disease and geographic atrophy in AMD). Ethnicity was categorized as Caucasian or Asian. The control subgroups were classified to population-based (PB) and hospital-based (HB).

### Statistical analysis

Based on the genotype frequencies for cases and controls, odds ratios (OR) with 95% confidence intervals (CI) were used to measure the strengths of associations. The statistical significance of the OR was determined with the *Z* test [35]. The heterogeneity assumption among studies was evaluated using a *χ*^2^-square-based *Q* test. If *P*-value > 0.10 for the *Q* test was indicated, a lack of heterogeneity among studies, other words, Mantel–Haenszel (fixed-effects model) was chosen, otherwise, the DerSimonian-Laird (random-effects model) was applied [36,37]. We investigated the correlation between rs10033900 and/or rs2285714 polymorphisms and AMD risk by testing whole five genetic models: A versus G, AG versus GG, AA + AG versus GG, AA versus GG and AA versus AG+GG. A sensitivity analysis was performed by omitting studies, one after another, to assess the stability of results. The departure of frequencies of the rs11200638 polymorphism from expectation under HWE was assessed by the Pearson’s *χ*^2^ test, *P* < 0.05 was considered significant [38]. The funnel plot was evaluated by Begg’s test, and the publication bias was evaluated by Egger’s test, whose *P*-value < 0.05 was considered significant [39]. All statistical tests for this meta-analysis were performed using version 10.0 Stata software (StataCorp LP, College Station, TX, U.S.A.). The power and sample size analysis of our meta-analysis was calculated by a program called PS: Power and Sample Size Calculation (http://biostat.mc.vanderbilt.edu/wiki/Main/PowerSampleSize#Windows).

### Network of gene-interaction of CFI gene

To more complete understanding of the role of CFI in AMD, the network of gene-gene interactions for CFI gene was utilized through String online server (http://string-db.org/) [40].

## Results

### Study searching and their basic information

Using various combinations of key terms, a total of 632 article titles were garnered by a document search using the PubMed (385 titles) and other databases (247 titles). As shown in Figure 1, 423 articles were excluded after screening the “Abstract” sections of the manuscripts. The full texts were then evaluated, and 198 additional articles were excluded due to duplication (154), meta-analysis or systematic analysis (28), only case group (4), and no data for each genotype (12). Finally, 11 different articles [23–33] were included in our meta-analysis, including 12 case–control studies about *CFI* gene rs10033900 polymorphism and total AMD risk and 3 case–control studies about rs2285714 polymorphism and AMD risk. The available clinical information in all publications were shown in Supplementary Table S1. Eleven case–control studies were involved to neovascular disease and geographic atrophy. All case–control studies about rs10033900 polymorphism were consistent with HWE in control groups (Table 1). In addition, we checked the minor allele frequency (MAF) reported for the six main worldwide populations in the 1000 Genomes Browser (https://www.ncbi.nlm.nih.gov/snp/rs10033900): Global (0.495), Europe (0.537), East Asian (0.388), South Asian (0.31), African (0.660), American (0.53) (https://www.ncbi.nlm.nih.gov/snp/rs2285714); Global (0.252), Europe (0.393), East Asian (0.202), South Asian (0.39), African (0.023), American (0.37) (Figure 2A,B). Finally, we calculated the C-allele frequency both in Asians and Caucasians in case and control groups, which suggested C-allele in Caucasians had higher frequency than Asians in both case and control groups (Figure 3). The genotyping methods included polymerase chain reaction-restrictive fragment length polymorphism and matrix-assisted laser desorption/ionization time-of-flight mass spectrometry, sequencing, mixed methods, and TaqMan.

**Figure 1:** Flow chart illustrating the search strategy used to identify association studies for *CFI* gene two polymorphisms and AMD risk

**Figure 2:** The MAF reported for the six main worldwide populations in the 1000 Genomes Browser The MAF of minor-allele (mutant-allele) for *CFI* gene rs10033900 (**A**) and rs2285714 (**B**) polymorphism from the 1000 Genomes online database and present analysis.

**Figure 3:** C-allele frequencies for the *CFI* gene rs10033900 polymorphism among cases/controls stratified by ethnicity

**Table 1:** Characteristics of included studies in *CFI* polymorphisms and AMD risk

Author	Year	Country	Ethnicity	Type	Case	Control	SOC	Cases			Controls			HWE	Genotype
								CC	CT	TT	CC	CT	TT		
rs1003900															
Total															
Yang	2014	China	Asian	Neovascular disease	300	299	HB	32	141	127	35	138	126	0.764	MALDI-TOF MS
Seddon	2010	U.S.A.	Caucasian	Advanced AMD	545	275	PB	120	278	147	87	134	54	0.852	MALDI-TOF MS
Reynolds	2009	U.S.A.	Caucasian	Advanced AMD	102	55	PB	29	50	23	20	28	7	0.561	MALDI-TOF MS
Cipriani	2012	U.K.	Caucasian	Advanced AMD	804	410	PB	186	407	211	101	207	102	0.843	Mixed methods
Cipriani	2012	U.K.	Caucasian	Advanced AMD	222	334	PB	45	130	47	80	177	77	0.273	Mixed methods
Wu	2013	China	Asian	AMD	235	140	HB	13	68	154	12	58	70	0.997	PCR-RFLP
Smailhodzic	2012	The Netherlands	Caucasian	Neovascular disease	192	144	HB	48	92	52	29	80	35	0.175	Sequencing
Aygun	2019	Turkey	Caucasian	Advanced AMD	109	92	HB	26	54	29	24	39	29	0.151	Sequencing
Qian	2014	China	Asian	AMD	288	384	HB	48	127	113	48	152	184	0.063	TaqMan
Kondo	2010	U.S.A.	Caucasian	Neovascular disease	116	189	HB	6	59	51	31	85	73	0.459	TaqMan
Peter	2011	U.S.A.	Caucasian	AMD	146	1260	PB	34	68	44	348	623	289	0.751	TaqMan
Yu	2011	U.S.A.	Caucasian	Advanced AMD	1072	216	PB	243	521	308	65	107	44	0.998	TaqMan
AMD type															
Seddon	2010	U.S.A.	Caucasian	Geographic atrophy	139	275	PB	26	72	41	87	134	54	0.852	MALDI-TOF MS
Reynolds	2009	U.S.A.	Caucasian	Geographic atrophy	53	55	PB	19	20	14	20	28	7	0.561	MALDI-TOF MS
Seddon	2010	U.S.A.	Caucasian	Neovascular disease	406	275	PB	94	206	106	87	134	54	0.852	MALDI-TOF MS
Reynolds	2009	U.S.A.	Caucasian	Neovascular disease	49	55	PB	10	30	9	20	28	7	0.561	MALDI-TOF MS
Yang	2014	China	Asian	Neovascular disease	300	299	HB	32	141	127	35	138	126	0.764	MALDI-TOF MS
Aygun	2019	Turkey	Caucasian	Geographic atrophy	46	92	HB	12	24	10	24	39	29	0.151	Sequencing
Smailhodzic	2012	The Netherlands	Caucasian	Neovascular disease	192	144	HB	48	92	52	29	80	35	0.175	Sequencing
Aygun	2019	Turkey	Caucasian	Neovascular disease	63	92	HB	14	30	19	24	39	29	0.151	Sequencing
Yu	2011	U.S.A.	Caucasian	Geographic atrophy	258	216	PB	56	121	81	65	107	44	0.998	TaqMan
Kondo	2010	U.S.A.	Caucasian	Neovascular disease	116	189	HB	6	59	51	31	85	73	0.459	TaqMan
Yu	2011	U.S.A.	Caucasian	Neovascular disease	814	216	PB	187	400	227	65	107	44	0.998	TaqMan
rs2285714															
Aygun	2019	Turkey	Caucasian	AMD	111	96	HB	42	56	13	32	47	17	0.971	Sequencing
Wu	2013	China	Asian	AMD	239	140	HB	124	111	4	68	71	1	<0.001	PCR-RFLP
Yang	2014	China	Asian	AMD	300	299	HB	188	92	20	167	121	11	0.052	MALDI-TOF MS

Abbreviations: HB, hospital-based; HWE, Hardy–Weinberg equilibrium of control group; MALDI-TOF MS, matrix-assisted laser desorption/ionization time-of-flight mass spectrometry; PB, population-based; PCR-RFLP, polymerase chain reaction followed by restriction fragment length polymorphism; SOC, source of control;.

### Quantitative synthesis

#### Rs10033900 polymorphism

In whole analysis, decreased associations were observed in three genetic models (C-allele vs. T-allele: OR: 0.87, 95% CI: 0.76–0.99, *P* = 0.001 for heterogeneity, Figure 4A, *P* = 0.029; CC vs. TT: OR: 0.75, 95% CI: 0.58–0.97, *P* = 0.003 for heterogeneity, *P* = 0.025; CC vs. CT+TT: OR: 0.82, 95% CI: 0.68–0.98, *P* = 0.039 for heterogeneity, *P* = 0.028). In subgroup analysis by ethnicity, based on different frequency of races, there had decreased associations between this polymorphism and AMD in Caucasians not Asians in all models (C-allele vs. T-allele: OR = 0.84, 95% CI = 0.77–0.91, *P*_heterogeneity_ = 0.125, *P* < 0.001, Figure 4B, CT vs. TT: OR = 0.87, 95% CI = 0.75–1.00, *P*_heterogeneity_ = 0.380, *P* = 0.047, CC+CT vs. TT: OR = 0.81, 95% CI = 0.70–0.92, *P*_heterogeneity_ = 0.246, *P* = 0.002, CC vs. TT: OR = 0.69, 95% CI = 0.54–0.88, *P*_heterogeneity_ = 0.060, *P* = 0.003; CC vs. CT+TT:OR = 0.77, 95% CI = 0.64–0.93, *P*_heterogeneity_ = 0.098, *P* = 0.007). In addition, regular analysis by source of control, also significantly trend were found for this SNP in PB rather than HB studies (C-allele vs. T-allele: OR = 0.82, 95% CI = 0.75–0.90, *P*_heterogeneity_ = 0.153, *P* < 0.001, CT vs. TT: OR = 0.84, 95% CI = 0.71–0.98, *P*_heterogeneity_ = 0.308, *P* = 0.031, Figure 5, CC+CT vs. TT: OR = 0.78, 95% CI = 0.67–0.91, *P*_heterogeneity_ = 0.159, *P* = 0.001, CC vs. TT: OR = 0.67, 95% CI = 0.56–0.81, *P*_heterogeneity_ = 0.173, *P* < 0.001; CC vs. CT+TT:OR = 0.76, 95% CI = 0.65–0.88, *P*_heterogeneity_ = 0.519, *P* < 0.001) (Table 2) (Figure 5). AMD have different types and stages, the difference of clinical presentation for dry and wet AMD is completely different, so we firmly believed that the correlations existed should be evaluated separately, significant negative associations were found both for geographic atrophy (such as C-allele vs. T-allele: OR = 0.72, 95% CI = 0.60–0.85, *P*_heterogeneity_ = 0.158, *P* < 0.001, CC vs. TT: OR = 0.51, 95% CI = 0.36–0.72, *P*_heterogeneity_ = 0.168, *P* < 0.001, Figure 6) and neovascular disease (for example in C-allele vs. T-allele: OR = 0.82, 95% CI = 0.74–0.91, *P*_heterogeneity_ = 0.237, *P* < 0.001, CC vs. TT: OR = 0.64, 95% CI = 0.51–0.80, *P*_heterogeneity_ = 0.142, *P* < 0.001, Figure 6). Finally, different genotype methods were applied in included studies, we tried to in each method, whether associations may exist in our analysis, we found some positive results in MALDI-TOF-MS (CC vs. CT+TT: OR = 0.69, 95% CI = 0.53–0.89, *P*_heterogeneity_ = 0.449, *P* = 0.004) (Figure 7) (Table 3).

**Figure 4:** Forest plot of AMD risk associated with *CFI* gene rs10033900 polymorphism (C-allele vs. T-allele) by ethnicity subgroup (**A**) Random effect model and (**B**) fixed effect model. The squares and horizontal lines correspond to the study-specific OR and 95% CI. The area of the squares reflects the weight (inverse of the variance). The diamond represents the summary OR and 95% CI.

**Figure 5:** Forest plot of AMD risk associated with *CFI* gene rs10033900 polymorphism (CT vs. TT) by source of control subgroup

**Figure 6:** Forest plot of AMD risk associated with *CFI* gene rs10033900 polymorphism (CC vs. TT) by AMD type subgroup

**Figure 7:** Forest plot of AMD risk associated with *CFI* gene rs10033900 polymorphism (CC vs. CT+TT) by genotyping methods subgroup

**Table 2:** Results of the meta-analysis on *CFI* polymorphisms and AMD risk in total and types of subgroups

Variables	*N*	Case/	C-allele vs. T-allele			CT vs. TT			CC+CT vs. TT			CC vs. TT			CC vs. CT+TT		
		Control	OR (95% CI)	*P*_h_	*P*	OR (95% CI)	*P*_h_	*P*	OR (95% CI)	*P*_h_	*P*	OR (95% CI)	*P*_h_	*P*	OR (95% CI)	*P*_h_	*P*
rs1003900																	
Total	12	4131/3798	0.87 (0.76–0.99)	0.001	0.029	0.89 (0.75–1.05)	0.040	0.177	0.85 (0.70–1.02)	0.004	0.073	0.75 (0.58–0.97)	0.003	0.025	0.82 (0.68–0.98)	0.039	0.028
Ethnicity																	
Asian	3	823/823	0.94 (0.62–1.41)	0.001	0.751	0.92 (0.58–1.52)	0.004	0.747	0.92 (0.54–1.57)	0.001	0.764	0.97 (0.51–1.82)	0.033	0.916	1.07 (0.79–1.45)	0.165	0.681
Caucasian	9	3308/2975	0.84 (0.77–0.91)	0.125	0.000	0.87 (0.75–1.00)	0.380	0.047	0.81 (0.70–0.92)	0.246	0.002	0.69 (0.54–0.88)	0.060	0.003	0.77 (0.64–0.93)	0.098	0.007
SOC																	
HB	6	1240/1248	0.93 (0.74–1.18)	0.002	0.549	0.96 (0.72–1.28)	0.027	0.781	0.94 (0.69–1.27)	0.009	0.668	0.86 (0.55–1.37)	0.013	0.532	0.89 (0.60–1.31)	0.026	0.548
PB	6	2891/2550	0.82 (0.75–0.90)	0.153	0.000	0.84 (0.71–0.98)	0.306	0.031	0.78 (0.67–0.91)	0.159	0.001	0.67 (0.56–0.81)	0.173	0.000	0.76 (0.65–0.88)	0.519	0.000
AMD type–																	
Neovascular disease	7	1940/1270	0.82 (0.74–0.91)	0.237	0.000	0.87 (0.73–1.04)	0.808	0.119	0.80 (0.68–0.95)	0.647	0.010	0.64 (0.51–0.80)	0.142)	0.000	0.72 (0.54–0.96)	0.068	0.024
Geographic atrophy	4	496/638	0.72 (0.60–0.85)	0.158	0.000	0.70 (0.52–0.95)	0.103	0.020	0.66 (0.42–1.04)	0.094	0.075	0.51 (0.36–0.72)	0.168)	0.000	0.66 (0.50–0.86)	0.355	0.003
Genotyping																	
Sequencing	2	301/236	1.05 (0.82–1.33)	0.962	0.707	0.97 (0.64–1.45)	0.176	0.876	1.01 (0.69–1.48)	0.339	0.974	1.10 (0.68–1.79)	0.956)	0.696	1.13 (0.75–1.69)	0.345	0.555
TaqMan	4	1622/2049	0.86 (0.63–1.17)	0.000	0.338	0.91 (0.65–1.28)	0.030	0.598	0.85 (0.57–1.27)	0.003	0.430	0.67 (0.35–1.28)	0.000)	0.223	0.75 (0.47–1.21)	0.006	0.239
MALDI-TOF MS	3	947/629	0.80 (0.69–0.93)	0.124	0.003	0.86 (0.68–1.10)	0.338	0.224	0.79 (0.63–1.00)	0.149	0.048	0.61 (0.45–0.83)	0.199)	0.002	0.69 (0.53–0.89)	0.449	0.004
Mixed methods	2	1026/744	0.95 (0.83–1.09)	0.886	0.474	1.02 (0.81–1.30)	0.371	0.846	0.98 (0.78–1.23)	0.472	0.890	0.90 (0.68–1.19)	0.912)	0.463	0.88 (0.70–1.11)	0.604	0.290
rs2285714																	
Total	3	650/535	1.13 (0.94–1.36)	0.833	0.210	0.72 (0.25–2.02)	0.063	0.527	0.86 (0.52–1.43)	0.107	0.564	0.92 (0.54–1.57)	0.178)	0.748	1.25 (0.99–1.58)	0.854	0.065

*P*_h_: value of *Q*-test for heterogeneity test; *P*: *Z*-test for the statistical significance of the OR

**Table 3:** Publication bias tests (Begg’s funnel plot and Egger’s test for publication bias test) for *CFI* rs1003900 and rs2285714 polymorphism

Egger’s test						Begg’s test	
Genetic type	Coefficient	Standard error	*t*	*P* value	95% CI of intercept	*z*	*P* value
**rs1003900**							
C-allele vs. T-allele	-2.336	2.042	−0.77	0.46	(−9.116–4.444)	0.62	0.537
CT vs. TT	-1.799	2.063	−0.87	0.404	(−6.396–2.798)	0.89	0.373
CC+CT vs. TT	-1.997	2.15	−0.93	0.375	(−6.788–2.793)	0.89	0.373
CC vs. TT	-0.994	1.16	−0.86	0.412	(−3.578–1.591)	0.48	0.631
CC vs. CT+TT	-0.577	1.243	−0.46	0.653	(−3.347–2.194)	0.62	0.537
**rs2285714**							
C-allele vs. T-allele	1.247	1.837	0.68	0.62	(−22.094–24.587)	0.52	0.602
CT vs. TT	-0.122	0.318	−0.38	0.767	(−4.168–3.923)	0.52	0.602
CC+CT vs. TT	-0.124	0.323	−0.38	0.766	(−4.234–3.985)	0.52	0.602
CC vs. TT	-0.092	0.321	−0.29	0.823	(−4.177–3.992)	0.52	0.602
CC vs. CT+TT	0.749	0.89	0.84	0.555	(−10.56–12.059)	0.52	0.602

#### Rs2285714 polymorphism

Given the limited case–control studies about this SNP, subgroups could not be analyzed separately. No association was detected in the whole data (data not shown) (Table 2).

### Bias diagnosis for publication and sensitivity analysis

The publication bias was evaluated by both Begg’s funnel plot and Egger’s test. At beginning, the shape of the funnel plots seemed asymmetrical in allele comparison for rs10033900 and rs2285714 by Begg’s test, suggesting no publication bias was existed. Then, Egger’s test was applied to provide statistical evidence of funnel plot symmetry. As a result, no obvious evidence of publication bias was observed (such as C-allele vs. T-allele, *t* = −0.77, *P* = 0.46 for Egger’s test; *z* = 0.62, *P* = 0.537 for Begg’s test, Figure 8A,B for rs10033900; C-allele vs. T-allele, *t* = 0.68, *P* = 0.62 for Egger’s test; *z* = 0.52, *P* = 0.602 for Begg’s test, Figure 8C,D for rs2285714) (Table 3).

**Figure 8:** The publication bias for CFI gene polymorphisms Begg’s funnel plot for publication bias test (C-allele vs. T-allele) (**A** for rs10033900; **C** for rs2285714). Each point represents a separate study for the indicated association. Log [OR], natural logarithm of OR. Horizontal line, mean effect size. Egger’s publication bias plot (C-allele vs. T-allele) (**B** for rs10033900; **D** for rs2285714).

To delete studies that may influence the power and stability of whole study, we applied the sensitive analysis, finally, no sensitive case–control studies were found for two SNPs (Figure 9A,B).

**Figure 9:** Sensitivity analysis for CFI gene polymorphisms Sensitivity analysis between CFI gene polymorphisms and AMD risk (C-allele vs. T-allele) (**A** for rs10033900; **B** for rs2285714).

### Gene–gene network diagram and interaction of online website

String online server indicated that CFI gene interacts with numerous genes. The network of gene–gene interaction has been illustrated in Figure 10.

**Figure 10:** Human CFI interactions network with other genes obtained from String server At least 10 genes have been indicated to correlate with HTRA1 gene. CFH: complement factor H; C3: complement C3; CFB: complement factor B; CD46: membrane cofactor protein; CFHR3: complement factor H-related protein 3; C4B: complement C4-B; C4A: complement C4-A; C2: complement C2; C4BPA: C4b-binding protein alpha chain; CR1: complement receptor type 1.

## Discussion

Because of the critical consequences about the visual loss caused by AMD, especially advanced AMD (atrophic/dry or neovascular/wet), it is necessary to study its etiology and mechanism, then to development early diagnostic methods and effective treatments. Nowadays, vascular endothelial growth factor (VEGF) inhibitors are widely recognized as effective drugs in clinical application for CNV (wet AMD) [41–43]. It is well known that VEGF is involved in wet AMD development because that the formation of angiogenesis and vascular permeability can lead to fluid leakage across the blood vessels, and visual loss in the final [44]. Anti-VEGF agents such as ranibizumab and bevacizumab have been widely applied in the clinic [45,46], in addition, have been proved to effectively slow the progress of CNV; however, heterogeneity was observed among patients in terms of the invalid samples and who have shorter duration of treatment [47]. It was hypothesized that genetic factors may participate in this period of this heterogeneous response, such as the variants of complement system genes. In addition, in the mechanism of dry AMD formation, inflammation and complement-mediated attack is existed in RPE, Bruch’s membrane and choroid region, which involves the complement cascade pathway. Increasing evidence has shown that inflammatory processes, especially the complement activation pathway, may play a major role in the pathogenesis of AMD [48,49]. Thus, we can regulate complement and inflammatory system to delay the development of dry AMD [50,51].

Next, to identify some novel detection markers and target drugs for different types of AMD is the current and future research focus on the direction. In the introduction section, we have enunciated the genetic factors may help us search potential high-risk group about AMD, which can be prevented and treated in advance. CFB, C2, C3, CFH in complement system has been widely reported. Another molecular CFI remains equivocal. Yang et al. made a meta-analysis that rs10033900 and rs2285714 SNPs had significant associations with AMD risk [32], whose report was indelicate that subgroups was not analyzed. An additional article in 2019 has been published, so we performed an updated meta-analysis to come to a more convincing conclusion about *CFI* gene polymorphisms and AMD susceptibility.

The best part of our analysis is that decreased associations were found about rs10033900 SNP and AMD risk in Caucasians, positive correlations were also observed both in geographic atrophy and neovascular disease subtype. In other words, if individuals carry on CC genotype or C-allele from peripheral blood test, which may indicate that it is possible to have a lower incidence of AMD, on the contrary, individuals carrying T-allele or TT genotype may have a high susceptibility for AMD. Therefore, it should offer us some preventions to intervene, or carry out treatments as soon as possible. To sum up, we wish to use this method to reduce the incidence of AMD and improve the cure rate of early treatment. In addition, the power of present study was 0.76, which suggested our conclusions were relative stable and convincing, which should be included more clinical information to confirm.

In addition, in order to identify the network correlation of CFI, the online analysis system-String was applied to predict potential and functional partners related to CFI, which can help us to better understand the value for detection and concern. Finally, ten genes were predicted. Among them, the scores are general high, and eight genes are members in complement system. In addition, researchers have focused on the complement pathways involved in AMD and their preventive/personalized medicine correspondingly [52,53].

The associations among AMD development and these genes majority involves gene polymorphisms. The highest score of association was CFH (0.999), Harrison et al. suggested the decreased heparin-binding affinity caused by the Y402H polymorphism (a common SNP in CFH gene) may recognize of SCR7^H402^, which may contribute to the pathogenesis of AMD [54]. C3 gene contains many SNPs, our previous meta and Zhang et al. both detected some increased and decreased SNPs in AMD [19,55]. Wang et al. performed a systematic analysis and suggested rs641153 in the CFB gene was a protective factor in advanced AMD both in Caucasians and Asians [17]. Rs547154 and rs9332739 SNPs had both decreased correlations to AMD risk [15]. In a word, we should deep explore these partners of CFI gene, and gene–gene interactions in the development of AMD in the next step.

There are some inherent limitations of our study should be declared. First, further studies should focus on Mixed and African populations, which was vacant in present analysis and need many more studies to consider rs2285714 SNP. Second, gene–gene and gene–environment interactions were not well analyzed. It is possible that specific environmental and lifestyle factors alter the associations between *CFI* polymorphisms and AMD, including age, diabetes, smoking, familial history and hypertension. Third, whether the AMD patients have other complications, such as kidney disease, heart disease, all the included paper have not been reported. Further comprehensive studies should include above information, which may influence the function of *CFI* gene polymorphisms. Fourth, vision is the most concerned-clinical indicator of AMD, future studies should include the value of the vision and analyze the relationships between *CFI* polymorphisms and the degree of visual impairment, which may help us better detect disease progression.

In conclusion, our present meta-analysis suggests that *CFI* rs10033900 polymorphism may be powerful associated with AMD risk, which may be as a clinical biomarker for detection in the future.

## Supplementary Material

Supplementary Table S1

## Abbreviations

AMD: age-related macular degenerative
CFI: complement factor I
CI: confidence intervals
HWE: Hardy–Weinberg equilibrium
OR: odds ratio
RPE: retinal pigment epithelium
VEGF: vascular endothelial growth factor
